RETRACTED

# Compound Ipratropium Bromide plus Budesonide Inhalation in the Treatment of Acute Exacerbation of Chronic Obstructive Pulmonary Disease and Its Effect on Heparin-Binding Protein

**DOI:** 10.1155/2022/4457740

**Published:** 2022-07-04

**Authors:** Yuan Dong, Qingling Li

**Affiliations:** China University of Mining and Technology, Xuzhou First People's Hospital, No. 269, Daxue Road, Tongshan, Xuzhou 221000, Jiangsu, China

## Abstract

**Objective:**

To analyze the clinical effect of compound ipratropium bromide combined with budesonide atomization inhalation on acute exacerbation of chronic obstructive pulmonary disease (AECOPD) and its effect on the heparin-binding protein.

**Methods:**

A total of 110 patients with AECOPD who were admitted to our hospital between January 2020 and January 2021 were enrolled and assigned into control group (conventional treatment + compound ipratropium bromide) and combined group (conventional treatment + compound ipratropium bromide + budesonide) in a 1 : 1 ratio according to different treatment methods. The clinical effects, pulmonary function indexes, and heparin-binding protein levels before and after treatment were compared between the two groups.

**Results:**

The treatment with oxygen-driven nebulization of ipratropium bromide combined with budesonide led to a significantly higher total effective rate versus the treatment with ipratropium bromide alone (*P* < 0.001). After treatment, remarkably higher arterial oxygen partial pressure (PaO_2_), arterial oxygen saturation (SaO_2_), forced vital capacity (FVC), forced expiratory volume in one second (FEV1), and FEV1/FVC in the combined group vs. the control group were observed (*P* < 0.001). The carbon dioxide partial pressure (PaCO_2_) levels in the two groups were significantly lower than those before treatment, and the decrease in the combined group was greater (*P* < 0.001). A significantl reduction was observed in heparin-binding protein in both groups after treatment, and the decrease in the combined group was greater versus the control group (*P* < 0.001).

**Conclusion:**

Compound ipratropium bromide plus budesonide via aerosol inhalation therapy might be a preferable approach for AECOPD patients. It exhibits a synergistic effect on inhibiting inflammatory mediators and cytokine networks, significantly reduces airway hyperresponsiveness, and improves blood gas indicators and lung function.

## 1. Introduction

Chronic obstructive pulmonary disease (COPD) is a common chronic inflammatory disease of the respiratory system [1]. The acute exacerbation of COPD (AECOPD) is characterized by incomplete reversible airflow, progressive development, and even respiratory failure due to airway constriction, increased mucus secretion, airflow restriction aggravation, and further ventilation dysfunction [2, 3]. The incidence has been on a rise and has become one of the leading causes of death worldwide. Statistics show that COPD is associated with persistent chronic cough and sputum, with a higher occurrence in over 40-year-old patients. If effective measures are not taken, it might develop into respiratory failure, pulmonary heart disease, and other diseases, constituting a worldwide public health concern [4]. Therefore, effective therapeutic strategies are urgent to counteract these rising trends. Compound ipratropium bromide is a commonly used drug for the treatment of AECOPD, which has the function of dilating bronchial tubes [5, 6]. Compound ipratropium bromide is a compound preparation of salbutamol and ipratropium bromide, in which salbutamol is a beta2 adrenergic receptor agonist and acts on all smooth muscles from the main trachea to the terminal alveoli, and has a strong bronchodilator effect. Nebulized budesonide is a glucocorticoid and has a high-efficiency local antiinflammatory effect. After entering the body through aerosol inhalation, it can inhibit immune response and reduce antibody synthesis. Reduce airway edema, improve lung function, and reduce the release and activity of allergic active mediators such as histamine, and its toxicity is weaker than other glucocorticoids [7, 8]. Compound ipratropium bromide is a potent anticholinergic drug with high selectivity for bronchial smooth muscle *M* receptors, and has a strong relaxation effect on bronchial smooth muscle. The combination of the two enhances the efficacy. In traditional Chinese medicine, AECOPD refers to the condition that the patient develops cough, shortness of breath, expectoration of sputum, wheezing, and increased sputum volume in a short period of time; it may be accompanied by systemic symptoms, such as fever. Chinese medicine believes that AECOPD belongs to the category of “lung inflation.” The main symptoms of acute exacerbation are “phlegm-dampness stagnation” and “lung hyperplasia.” In this study, Chinese medicine adjuvant therapy was used to obtain good clinical efficacy. The principal objective of this study is to determine the efficacy of compound ipratropium bromide plus budesonide nebulizer inhalation on AECOPD.

RETRACTED

## 2. Materials and Methods

### 2.1. Patients

A total of 110 patients with AECOPD who were admitted to our hospital between January 2020 and January 2021 were enrolled and assigned into control group and combined group in a 1 : 1 ratio according to different treatment methods. The control group included 36 males and 19 females, aged 47 to 79 years, with an average age of 57.34 ± 15.72 years, and the duration of COPD was 5 to 20 years, with an average duration of 9.55 ± 3.24 years. The combined group included 34 males and 21 females, aged 49 to 80 years, with an average age of 58.01 ± 14.62 years, and the duration of COPD was 4 to 21 years, with an average course of 9.79 ± 3.84 years. The baseline profile such as gender, age, and course of disease in the two groups were balanced.

This study was approved by the Medical Ethics Committee of the Affiliated Hospital of China Mining University, No. #297/116, and the patients were informed of the contents of this study and signed informed consent.

### 2.2. Inclusion and Exclusion Criteria

Inclusion criteria: (1) met the diagnostic criteria for COPD in the Guidelines for the Diagnosis and Treatment of Chronic Obstructive Pulmonary Disease; (2) in acute exacerbation stage, presenting severe shortness of breath, combined with wheezing chest tightness, dyspnea, changes in sputum volume, color and viscosity, cough worsening, etc.; and (3) the patient did not choose other drugs for atomization treatment within 1 week. Exclusion criteria: (1) patients with long-term use of glucocorticoids; (2) patients with contraindication to the use of glucocorticoids; (3) patients with other lung diseases; (4) patients with severe heart, liver, kidney, endocrine and metabolic systems, and mental disorder; and (5) patients with active peptic ulcer, cataract, glaucoma, and other diseases.

### 2.3. Methods

Both groups of AECOPD patients were given basic treatment, including expectorant, antiinfection, oxygen therapy, and water and electrolyte balance. At the same time, Jianfei decoction was used for supporting treatment. The drug composition was licorice 15 g, pinellia 17 g, angelica 13 g, asarum 18 g, schisandra 14 g, silkworm 10 g, radish 10 g, and calamus 10 g. The above medicines are decocted with water, 1 dose a day, 2 times in the morning and evening.

The patients in the control group were treated with aerosol inhalation of compound ipratropium bromide on the basis of basic treatment and supporting treatment: 1.25 mL of compound ipratropium bromide solution (Shanghai Boehringer Ingelheim Pharmaceutical Co., Ltd., approval number: H20050296) was inhaled and continuously pressurized via aerosol inhalation, at an oxygen flow of 6–8 L per minute, 5–10 min each time, once every two days; one treatment course was taken as 7 d.

The patients in the combined group were treated with oxygen-driven nebulization of ipratropium bromide combined with budesonide via inhalation of compound suspension (Alikang Pharmaceutical Co., Ltd., approval number: H20090903): 1.25 mL of inhaled compound ipratropium bromide solution and 0.5 mg of inhaled budesonide device were used for continuous pressurized aerosol inhalation treatment, at an oxygen flow of 6–8 L/min, 5–10 min each time, once every two days; one treatment course was taken as 7 d. The mitigation of symptoms and clinical data of the two groups were observed and the curative effect was evaluated.

RETRACTED

### 2.4. Outcomes

(1) Clinical efficacy. TCM symptoms and signs were combined to calculate the score [9], and the clinical efficacy was determined by the change rate of the score.
  (1) $$\begin{array}{c} \text{Change rate of points}=\frac{\left(\text{points before treatment}-\text{points after treatment}\right)}{\text{points before treatment}}\times 100\%. \end{array}$$
Markedly effective: dyspnea disappeared completely, cough and sputum were significantly reduced, wet squeaks and wheezing sounds completely disappeared, and the white blood cell count returned to normal point reduction rate ≥80%; effective: dyspnea was improved to some extent, the cough was relieved, the sputum volume was reduced, the chirp sound was relieved, and the white blood cell count decreased, 70% ≤ point reduction rate < 80%; ineffective: no change or aggravation of dyspnea, increased sputum volume, aggravated chirp sound, and no change or increase in white blood cell count, point reduction rate <70%.
  (2) $$\begin{array}{c} \text{Total effective rate}=\frac{\left(\text{markedly effective}+\text{effective}\right)}{\text{total number of cases}}\times 100\%. \end{array}$$
(2) Blood gas index. Arterial oxygen partial pressure (PaO_2_), arterial oxygen saturation (SaO_2_), and carbon dioxide partial pressure (PaCO_2_) were measured and compared. The blood gas index was tested by a 348EX blood gas analyzer (manufacturer: Siemens Medical Diagnostic Products Co., Ltd., registration number: State Food and Drug Administration Equipment (Jin) 2014 No. 2402991). Hospital testing personnel were trained for equipment standard operation, and all items were tested in accordance with the instructions.
(3) Pulmonary function indexes. The forced vital capacity (FVC) and forced expiratory volume in one second (FEV1) were measured by a spirometer, and the FEV1/FVC value was calculated.
All the tested patients stopped taking hormonal drugs 48 hours before the pulmonary function test, stopped taking bronchodilators 24 hours before the examination, stopped taking bronchodilator aerosol 12 hours before the examination, and smoked 72 hours before the examination. The basal lung function, including FVC and lung volume, was measured first. Each item was measured 3–5 times, with the optimal 3 times having a comparison error of ≤5%; then 200 mcg of bronchodilator Chuanloning aerosol was inhaled, and then FVC was measured after 10 minutes. The predicted value of FEV1% cannot be recovered to the 80% selected for this study. Except for FEV1/FVC, which is expressed as the ratio of the measured value, the remaining data, including FVC and FEV1, are expressed as the percentage of the measured value to the predicted value. The instrument used was the American Sensor Medics 2100 automatic computerized lung function tester.
(4) Changes of heparin-binding protein (HBP). Venous blood samples were collected from the patients within 24 hours of admission, and plasma samples were collected after centrifugation. The Jet-iStsr3000 immunofluorescence analyzer (Zhonghan Shengtai Biotechnology Co., Ltd., Zhejiang, China) was used to detect HBP by immunofluorescence.

RETRACTED

### 2.5. Statistical Analysis

Data were expressed as the mean ± standard deviation and cases (%). Statistical analysis was performed using the SPSS 22.0 (IBM, Armonk, NY, USA). Differences between groups were compared using Student's *t*-test and chi-square test, respectively. All statistical significance levels were set at a *P* value of less than 0.05.

## 3. Results

### 3.1. Clinical Efficacy

The treatment with oxygen-driven nebulization of ipratropium bromide combined with budesonide led to a significantly higher total effective rate versus the treatment with ipratropium bromide alone (94.54% vs. 72.73%) (*P* < 0.001), as shown in Table 1.

### 3.2. Blood Gas Indexes and Pulmonary Function Indexes

There was no significant difference in blood gas and pulmonary function indexes between the two groups before treatment (*P* > 0.05). After treatment, remarkably higher PaO_2_, SaO_2_, FVC, FEV1, and FEV1/FVC in the combined group vs. the control group were observed (*P* < 0.001), the PaCO_2_ levels in the two groups were significantly lower than those before treatment, and the decrease in the combined group was greater (*P* < 0.001), as shown in Table 2.

### 3.3. Changes of Heparin-Binding Protein

A significant reduction was observed in heparin-binding protein in both groups after treatment, and the decrease in the combined group was greater versus the control group (*P* < 0.001), as shown in Table 3.

## 4. Discussion

AECOPD features a long disease course and repeated attacks and is associated with respiratory muscle atrophy, declined pulmonary ventilation function, respiratory failure, and weakened immune function, which necessitates an alternative drug to overcome the undesirable results [9, 10].

Compound ipratropium bromide is a compound preparation of two bronchodilator drugs, salbutamol and ipratropium bromide, in which salbutamol is a *β*2 adrenergic receptor agonist, which acts on all smooth muscles from the main trachea to the terminal alveoli, and has a strong bronchodilator effect [11]. Ipratropium bromide is an anticholinergic drug with high selectivity for *M* receptors of bronchial smooth muscle. It can relax bronchial smooth muscle, reduce mucus secretion and tissue edema, and has little impact on respiratory glands and the cardiovascular system [12–14]. Reportedly, it can promote the ciliary movement of the bronchial mucosa and facilitate the discharge of sputum [15]. The two are confined to the lungs after inhalation and can jointly enhance the efficacy of the drug. Hormone therapy is of great significance due to the inflammatory response of acute exacerbation of the disease, but systemic use of hormones has been limited in clinical treatment due to its poor safety [16]. As an adrenal cortex hormone, budesonide can enhance the transcription process of *β*2 receptor protein on the cell membrane of patients' lung tissue, enhance the cooperation of respiratory mucosal receptor protein, reduce receptor affinity, and minimize down-regulation. The release can be significantly inhibited, reducing airway resistance and airway obstruction, thereby effectively relieving a series of symptoms such as chest tightness, shortness of breath, and dyspnea in patients [17, 18]. Traditional Chinese medicine believes that AECOPD is phlegm-dampness obstructing the lungs, and qi stagnation occurs in the chest, so symptoms such as cough, wheezing, excessive phlegm, and shortness of breath appear [7]. The licorice in the Jianfei recipe used in this study has the effect of removing phlegm and relieving cough. The main effect of Pinellia is to dry dampness and phlegm. The main effect of Angelica is to relieve lung orifice, asthma, and cough. Asarum warms the lung and resolves cough and asthma due to insufficiency of the kidneys. Bombyx batryticatus is flat in nature and has the effect of resolving phlegm and dispersing knots. Radix is pungent and sweet, mainly used for eliminating phlegm and relieving cough in chronic bronchitis. Calamus is warm in nature, bitter in taste, and can relieve spasm. Modern pharmacology believes that the active ingredient in licorice is licorice flavonoids, which can be antiinflammatory; licorice can also promote the secretion of respiratory mucosa, making it easy to cough up phlegm. Angelica imperatorin, an active ingredient in white peony root, can inhibit tumor necrosis factor-*a* in inflammatory tissues to achieve anti-inflammatory purposes. Schisandra can enhance the function of bronchial epithelial cells. These drugs can be used in combination to expel phlegm and relieve cough, and enhance lung function.

RETRACTED

According to the results of this study, the oxygen-driven nebulization of ipratropium bromide plus budesonide is associated with a higher total effective rate versus ipratropium bromide alone, suggesting that the compound ipratropium bromide combined with budesonide has a good efficacy profile in the treatment of AECOPD. Additionally, we found that after treatment, the oxygen-driven nebulization of ipratropium bromide plus budesonide resulted in a higher PaO_2_, SaO_2_, FVC, FEV1, and FEV1/FVC, but a lower PaCO_2_, indicating that the combination of the two inhibits the generation of inflammatory substances, shrinks and expands mucosal blood vessels via their action on lung tissues. Therefore, in addition to rational drug use and oxygen inhalation therapy, the use of compound ipratropium bromide plus budesonide for aerosol inhalation in the treatment of AECOPD patients can effectively regulate the patients' airway obstruction and improve the their blood gas indexes and lung function [19, 20]. HBP is a proinflammatory protein secreted by neutrophils. When infection occurs, bacteria or bacterial metabolites stimulate neutrophils to produce HBP, resulting in increased HBP levels in the body [21]. Paulsson [22] pointed out that serum PCT and HBP levels in patients with acute respiratory tract infection were significantly higher than those in healthy controls, which may be new biomarkers for the diagnosis of respiratory tract infection. The results of this study showed that after treatment, the levels of HBP in both groups decreased significantly, and the decrease was greater in the combined group. This finding suggests a promising outcome in inhibiting the release of inflammatory mediators and reducing the inflammatory response in patients.

Taken together, compound ipratropium bromide plus budesonide via aerosol inhalation therapy might be a preferable approach for AECOPD patients. It exhibits a synergistic effect on inhibiting inflammatory mediators and cytokine networks, significantly reducing airway hyperresponsiveness, and improving blood gas indicators and lung function. It is worth noting that it features smaller dosage aerosol inhalation, faster action, the property of being user-friendly, fewer side effects, and direct action on the lesion site.

## Figures and Tables

**Table 1:** Clinical efficacy.

Groups	*n*	Markedly effective	Effective	Ineffective	Total (%)
Combined group	55	42	10	3	52 (94.54)
Control group	55	14	26	15	40 (72.73)
*X* ^2^					10.031
*P*					<0.001

**Table 2:** Comparison of blood gas indexes and pulmonary function indexes in two groups of patients (*x* ± *s*).

Groups	*N*	PaO_2_ (mmHg)		SaO_2_ (%)		PaCO_2_ (mmHg)		FVC (L)		FEV1 (%)		FEV1/FVC (%)	
		Before	After	Before	After	Before	After	Before	After	Before	After	Before	After
Combined group	55	48.64 ± 3.75	70.06 ± 7.85	53.79 ± 6.84	66.28 ± 6.48	73.51 ± 5.68	42.51 ± 4.77	1.63 ± 0.27	3.66 ± 0.74	0.77 ± 0.23	1.99 ± 0.32	48.67 ± 5.46	62.49 ± 7.34
Control group	55	48.37 ± 3.96	62.31 ± 6.03	52.97 ± 6.39	57.29 ± 4.88	72.87 ± 5.07	48.16 ± 4.28	1.65 ± 0.24	2.89 ± 0.61	0.76 ± 0.22	1.60 ± 0.25	48.69 ± 5.28	56.18 ± 6.72
*t*		0.367	5.806	0.65	8.219	0.682	6.538	0.259	3.667	0.354	2.337	0.594	10.428
*P*		0.714	<0.001	0.517	<0.001	0.497	<0.001	0.487	<0.001	0.618	<0.001	0.529	<0.001

RETRACTED

**Table 3:** Changes of heparin-binding protein levels before and after the treatment in two groups of patients (*x* ± *s*).

Groups	*n*	HBP (ng/mL)	
		Before	After
Combined group	55	55.73 ± 12.67	14.38 ± 4.52
Control group	55	57.34 ± 11.95	21.39 ± 5.67
*T*		0.686	7.17
*P*		0.494	<0.001

## Data Availability

No data were used to support this study.
